The article "miR-221/222 promote tumor growth and suppress apoptosis by targeting lncRNA GAS5 in breast cancer" was retracted in 2021. Reasons: duplicated images; original data or images not available.

# miR-221/222 promote tumor growth and suppress apoptosis by targeting lncRNA GAS5 in breast cancer

**DOI:** 10.1042/BSR20181859

**Published:** 2019-01-15

**Authors:** Yuanyuan Zong, Yazhou Zhang, Xichao Sun, Tao Xu, Xiankui Cheng, Yejun Qin

**Affiliations:** 1 Department of Pathology, Shandong Provincial Hospital Affiliated to Shandong University, Jinan, Shandong 250021, P.R. China; 2 Department of Gastrointestinal Surgery, Shandong Provincial Hospital Affiliated to Shandong University, Jinan, Shandong 250021, P.R. China

**Keywords:** apoptosis, breast cancer, GAS5, miR-221/222

## Abstract

MicroRNAs (miRNAs) are 21–23-nucleotide, short, non-coding RNAs that play important roles in virtually all biological pathways in mammals and other multicellular organisms. The association of miR-221 and miR-222 (miR-221/222) for breast cancer is critical, but their detailed roles in its development and progression remain unclear. In the present study, we found that miR-221/222 were consistently up-regulated in breast cancer tissues. We then investigated the molecular mechanisms by which miR-221/222 contributed to breast cancer and identified growth arrest–specific transcript 5 (GAS5) as a direct target gene of miR-221/222. In contrast with the up-regulated expression levels of miR-221/222, GAS5 levels were significantly down-regulated and negatively correlated with miR-221/222 in breast cancer tissues. In addition, we showed that miR-221/222 inhibitors increased cellular apoptosis, miR-221/222 mimics decreased the cell apoptosis in breast cancer cells, and restoration of GAS5 expression attenuated the anti-apoptotic effects of miR-221/222 in breast cancer cells, indicating that GAS5 was a direct mediator of miR-221/222 function. Finally, we showed that miR-221/222 suppressed GAS5 expression significantly and enhanced tumor growth in a mouse model of breast cancer xenografts. The present study highlighted the important role of miR-221/222 as oncomiRs in breast cancer, which inhibited GAS5 translation. These findings may provide a new perspective for the molecular mechanism of breast carcinogenesis and provide a novel approach to the treatment of breast cancer.

## Introduction

Growth arrest–specific transcript 5 (GAS5), which is a long non-coding RNA (lncRNA), is a tumor-suppressor gene located on 1q25.1. It was initially found to bind to the glucocorticoid response element on the glucocorticoid receptor and inhibit DNA transcription induced by the glucocorticoid receptor [1]. Recently, several studies have reported that GAS5 expression is decreased in various tumor types, including prostate cancer [2], lung cancer [3], bladder cancer [4], liver cancer [5], colon cancer [6], pancreatic cancer [7], and breast cancer [8]. Most cellular studies have shown that GAS5 is mainly involved in regulating the apoptosis of tumors. Recently, Zhang et al. [9] reported that miR-21 negatively regulated GAS5 in its role in cancer progression. In addition, GAS5 also inhibits protein synthesis and regulates lymphocyte proliferation by regulating the mTOR signaling pathway in PC cells [10]. However, the exact mechanisms of GAS5 in breast cancer remain complex and obscure.

MicroRNAs (miRNAs) have opened new prospects for molecular research in breast cancer [11]. In recent years, the functional study of miR-221/222 in breast cancer has made it possible for miR-221/222 to become a molecular biomarker in breast cancer. miR-221/222 have high homology and play a biological role as an miR-221/222 cluster [12]. Studies have found that miR-221/222 play an oncogenic role in breast cancer. The target gene discovered at the earliest stage of miR-221/222 is the cell cycle-dependent protein kinase inhibitor, p27kip1 [13]. miR-221/222 exert a cancer-promoting effect by inhibiting this inhibitor. In recent years, it has been found that miR-221/222 have a higher expression level in triple-negative breast cancer and promote malignant tumor progression by targeting the negative regulation of TRPS1 [14]. Therefore, miR-221/222 are expected to become a new target for future breast cancer treatment.

In the present study, we found that miR-221/222 levels were consistently up-regulated in breast cancer tissues. Subsequently, we showed that miR-221/222 enhanced tumor growth in a breast cancer xenograft mouse model. Furthermore, we identified potential target genes of miR-221/222 and found that miR-221/222 inhibited the apoptosis of breast cancer cells by directly targeting an important tumor suppressor, GAS5.

## Materials and methods

### Human tissues and cell lines

A total of 48 pairs of breast cancer tissues and normal adjacent tissues were collected from patients at the Provincial Hospital Affiliated to Shandong University (Jinan, China) and written informed consent was get from each patient. After resection, tissue fragments were immediately frozen in liquid nitrogen and then stored at −80°C. The human breast cancer cell lines (MCF-7, MDA-MB-231, MDA-MB-453, and SKBR3) and the normal breast mammary epithelial cell line MCF-10A were purchased from the Shanghai Cell Bank of the Chinese Academy of Sciences (Shanghai, China). The cells were maintained in DMEM medium supplemented with 10% fetal bovine serum (FBS, Gibco, U.S.A.) at 37°C under 5% CO_2_ water-saturated atmosphere.

### RNA extraction and quantitative RT-PCR

Total RNA from the human tissues and culture cells was extracted using Trizol reagent following the protocols. The total RNA concentration was determined using a BioPhotometer (Eppendorf, Germany). qRT-PCR was performed on an Applied Biosystems 7500 Fast Real-Time PCR systems (Applied Biosystems). GAPDH and U6 were used as endogenous controls for GAS5 and miR-221/222, respectively. The sequences of the primers were as follows: GAS5 (sense): 5′-GAG AGT GGT GTG GGG AAC TG-3′; GAS5 (antisense): 5′-CAG AGG TCC CAC TGC ATG TT-3′; GAPDH (sense): 5′-TTG TCAA GCT CGT TTC TTG GT-3′; and GAPDH (antisense): 5′-CCT AGT CTC CAT GGT CTC ACT-3′. miR-221 (sense): 5′-ACA CTC CAG CTG GGA GCT ACA TTG TCT GCT GG-3′; and miR-221 (antisense): 5′-CTC AAC TGG TGT CGT GGA-3′; miR-222 (sense): 5′-ACA CTC CAG CTG GGA GCT ACA TCT GGC TAC TG-3′; and miR-222 (antisense): 5′-CTC AAC TGG TGT CGT GGA-3′; U6 (sense): 5′-CTC GCT TCG GCA GCA CA-3′; and U6 (antisense): 5′-AAC GCT TCA CGA ATT TGC GT-3′.

### Knockdown or overexpression of miR-221/222

Knockdown or overexpression of miR-221/222 was achieved by transfection with miRNA inhibitors or miRNA mimics. Synthetic miR-221/222 mimics (pre-miR-221/222), inhibitors (antimiR-221/222), and scrambled negative control RNAs (pre-miR-control and anti-miRcontrol) were purchased from GenePharma (Shanghai, China). MCF-7, MDA-MB-231, and SKBR3 cells were seeded in six-well plates using RPMI 1640 medium supplemented with 10% FBS. The cells were transfected with Lipofectamine 2000 (Invitrogen, Thermo Fisher Scientific, Inc.) according to the manufacturer’s protocol. For each well, equal amounts of pre-miR-221/222, pre-miR-control, anti-miR-221/222, or anti-miRcontrol were used. After 6 h, the medium was changed to RPMI 1640 supplemented with 2% FBS. The cells were collected at 24 or 48 h after transfection and used for subsequent analysis.

### SiRNA interference and plasmid construction

SiRNA sequence targeting the human GAS5 cDNA was designed and synthesized by Ribobio (Guangzhou, China). The siRNA sequence was as follows: 5′-CUU GCC UGG ACC AGC UUA AUU-3′. A scrambled siRNA was synthesized as a negative control. A mammalian expression plasmid encoding the full-length human GAS5 open reading frame (ORF) without the miR-221/222-responsive 3′-UTR was purchased from Invitrogen. An empty plasmid was used as the negative control. The GAS5 siRNA and the GAS5 expression plasmid were transfected into MCF-7 cells using Lipofectamine 2000 (Invitrogen, Thermo Fisher Scientific, Inc.) according to the manufacturer’s instructions. Total RNA were isolated 24 h post-transfection. The GAS5 mRNA expression levels were assessed by quantitative RT-PCR.

### Luciferase reporter assays

The entire 3′-UTR of the human GAS5 transcript was amplified by PCR using human genomic DNA as a template. The PCR products were inserted into the p-MIR-reporter plasmid (Ambion, Austin, TX, U.S.A.). To test the binding specificity, the sequences that interact with the miR-221/222 seed sequence were mutated, and the mutant GAS5 3′-UTR was inserted into an equivalent luciferase reporter. For the luciferase reporter assay, HEK293T cells were cultured in 24-well plates. After 48 h, the cells were lysed and luciferase expression was measured using the Dual-luciferase assay system (Promega, U.S.A.) following the manufacturer’s protocol. The renilla luciferase (Rluc) was normalized by the firefly luciferase (Luc).

### Flow cytometric assay

The apoptosis of MCF-7 cells was examined using flow cytometry. After transfection for 48 h, cells were collected in the log phase of growth and the apoptotic cells were identified using an Annexin-V-FLUOS Staining kit (Roche Diagnostics GmbH). After washing with cold PBS, the cells were resuspended in binding buffer followed by staining with Annexin V-FITC/PI for 15 min in the dark at room temperature. The fluorescence signals were collected by FACSCanto (BD Bioscience, San Jose, CA) and then analyzed by FlowJo 8.7.1 software (Ashland, OR).

### Establishment of tumor xenografts in mice

Four-week-old female BALB/c nude mice were purchased from the Shanghai SLAC Laboratory Animal Co., Ltd, China. MCF-7 cells were infected with a control lentivirus or lentiviruses to overexpress miR-221 or miR-222. After infection and transfection, MCF-7 cells were subcutaneously injected into xenograft mice (1 × 10^7^ cells per mouse). The mice were killed after 25 days. The tumor xenografts were removed and taken photo, followed by measuring the weight of the tumors. Parts of the tumors were used for total RNA extraction, and the remaining tumors were fixed in 4% neutral-buffered formalin for hematoxylin and eosin (H&E) staining or Ki67 staining.

### Statistical analysis

The data were presented as mean ± SD of at least three independent experiments. The differences were considered statistically significant at *P*<0.05 using Student’s *t*-test. Prism 5.0 software (GraphPad, Inc., La Jolla, CA, U.S.A.) was used for data analyzes.

## Results

### miR-221/222 are up-regulated and GAS5 is down-regulated in breast cancer tissues and cell lines

In the first, the expression levels of miR-221/222 in 48 pairs of breast cancer tissues and normal adjacent were identified by quantitative RT-PCR. We found that miR-221/222 levels were consistently increased in breast cancer tissues compared with non-cancerous tissues (Figure 1A,B). In addition, there was a decreased expression of GAS5 in human breast cancer tissues compared with the normal adjacent tissues (Figure 1C).

**Figure 1:** Expression levels of miR-221/222 in breast cancer tissues (**A** and **B**) Quantitative RT-PCR analysis of the individual alteration of miR-221/222 in 48 pairs of breast cancer tissue (tumor) compared with matched normal adjacent tissue (normal) samples. (**C**) Quantitative RT-PCR analysis of the mean expression levels of GAS5 in 48 pairs of breast cancer tissue (tumor) and matched normal adjacent tissue (normal) samples. Each bar represents the mean ± SD values.

### Validation of GAS5 as a direct target of miR-221/222

To explore the molecular mechanism by which miR-221/222 contributes to breast cancer progression, starBase and Genome Browser were used in combination to search for potential targets of miR-221/222 (Figure 2). The correlation between miR-221/222 and GAS5 was further investigated in three human breast cancer cell lines, MCF-7, MDA-MB-231 and SKBR3, after overexpression or knockdown of miR-221/222. As expected, cellular miR-221/222 levels were significantly increased when MCF-7, MDA-MB-231 and SKBR3 cells were transfected with miR-221/222 mimics and were decreased when treated with miR-221/222 antisenses (Figure 3A). Therefore, the introduction of miR-221/222 mimics in MCF-7, MDA-MB-231 and SKBR3 cells significantly reduced the GAS5 expression, whereas miR-221/222 antisenses remarkably increased the GAS5 mRNA levels (Figure 3B). Then, a luciferase reporter assay was performed to confirm that miR-221/222 directly target the presumed binding site in the GAS5 3′-UTR and negatively regulate GAS5 expression. The GAS5 3′-UTR containing the presumed miR-221/222 binding site was fused downstream of the firefly luciferase gene in a reporter plasmid. The recombination plasmid was co-transfected into HEK293T cells along with miR-221/222 mimics. The mutated luciferase reporter was unaffected by overexpression of miR-221/222 (Figure 3C). This finding suggested that miR-221/222 directly bind to the 3′-UTR of the GAS5 transcript to inhibit the expression of GAS5.

**Figure 2:** GAS5 was a direct target of miR-221/222. starBase and Genome Browser were used to predict GAS5 as a target of miR-221/222

**Figure 3:** GAS5 was a direct target of miR-221/222 (**A** and **B**) Quantitative RT-PCR analysis of miR-221/222 levels in MCF-7, MDA-MB-231 and SKBR3 cells transfected with equal doses of premiR-221/222, anti-miR-221/222 or scrambled negative control RNAs (pre-miR-control or anti-miR-control). (**C**) Firefly luciferase reporters containing either wild-type (WT) or mutant (MUT) miR-221/222 binding sites in the GAS5 3′-UTR were co-transfected into HEK293T cells along with equal doses of pre-miR-221/222 or pre-miR-control. The cells were assayed using a luciferase assay kit 24 h post-transfection. Firefly luciferase values were normalized to β-gal activity, and the results were calculated as the ratio of firefly luciferase activity in the miR-221/222-transfected cells normalized to the premiR-control-transfected cells; **P<0.01; ***P<0.001.

### miR-221/222 suppress apoptosis in breast cancer cells by inhibiting GAS5

As a well-known pro-apoptotic gene, GAS5 was investigated to determine whether it can silence miR-221/222 to suppress breast cell apoptosis via flow cytometry. The results showed that the percentage of apoptotic cells in transfected with miR-221/222 mimics group was significantly lower. Moreover, there were a higher percentage of apoptotic cells after transfection with miR-221/222 antisenses (Figure 4A). Therefore, it was suggested that miR-221/222 function as anti-apoptotic factors in breast cancer cells. Next, we investigated whether miR-221/222 may regulate the apoptosis of breast cancer cells through a GAS5-dependent manner. In the first, we found the cells transfected with miR-221/222 mimics plus GAS5-overexpression plasmid exhibited a significantly higher GAS5 mRNA level compared with cells transfected with miR-221/222 mimics plus control plasmid (Figure 4B), suggesting that the overexpression of miR-221/222-resistant GAS5 was sufficient to rescue the suppression of GAS5 by miR-221/222. Moreover, MCF-7 cells simultaneously transfected with miR-221/222 mimics and the GAS5-overexpression plasmid showed significantly higher apoptotic rates than the cells transfected with miR-221/222 mimics plus control plasmid, indicating that the overexpression of miR-221/222-resistant GAS5 was sufficient to attenuate the anti-apoptotic effects of miR-221/222.

**Figure 4:** Effects of miR-221/222 and GAS5 on the apoptosis of breast cancer cells (**A**) Apoptosis assays were performed 24 h after the transfection of MCF-7 cells with equal doses of pre-miR-221/222, anti-miR-221/222 or scrambled negative control RNAs (pre-miR-control or anti-miR-control), or with equal doses of pre-miR-control plus control plasmid, pre-miR-221/222 plus control plasmid, pre-miR-control plus GAS5-overexpression plasmid or pre-miR-221/222 plus GAS5-overexpression plasmid. (**B**) Quantitative RT-PCR analysis of GAS5 mRNA levels in MCF-7 cells transfected with equal doses of pre-miR-control plus control plasmid, premiR-221/222 plus control plasmid, pre-miR-control plus GAS5-overexpression plasmid or pre-miR-221/222 plus GAS5-overexpression plasmid. *P<0.05; **P<0.01; ***P<0.001.

### miR-221/222 function as oncomiRs in breast cancer

Next, a xenograft mouse model was used to evaluate the biological effects of miR-221/222. MCF-7 cells (control lentivirus or lentiviruses to overexpress miR-221 or miR-222) were subcutaneously implanted into 4-week-old nude mice, and the mice were executed at day 25 after cell implantation. We found that the size and weight of tumors were significantly increased in the miR-221/222-overexpressing group compared with the control group (Figure 5A,B). Subsequently, we detected the expression levels of miR-221/222 in the tumor tissues and determined the miR-221/222-overexpressing significantly increased in miR-221/222 expression compared with tumors from the control group (Figure 5C).

**Figure 5:** Effects of miR-221/222 on tumor growth in a breast cancer xenograft mouse model (**A**) MCF-7 cells were infected with a control lentivirus or lentiviruses to overexpress miR-221 or miR-222. After infection, MCF-7 cells (1 × 10^7^ cells per 0.1 ml) were subcutaneously implanted into 4-week-old nude mice (eight mice per group), and tumor growth was evaluated on day 25 after cell implantation. Representative images of the tumors from the implanted mice. (**B**) Quantitative analysis of the tumor weights. (**C**) Quantitative RT-PCR analysis of miR-221/222 levels in the tumors from implanted mice. (**D**) Quantitative RT-PCR analysis of GAS5 mRNA levels in the tumors from implanted mice. (**E**) Representative H&E-stained and Ki-67-stained sections of the tumors from implanted mice; *P<0.05; **P<0.01.

Next, we found a reduced GAS5 mRNA levels in the tumors from the mice infected with miR-221/222 overexpressing MCF-7 cells compared with tumors from the control group (Figure 5D). Furthermore, H&E staining of tumor tissues revealed more cell mitosis in the miR-221/222-overexpressing groups compared with the control group. Finally, the proliferation activity of the tumor cells was assessed via Ki67 staining. The tumor cell proliferation rate was increased in tumors from the miR-221/222-overexpressing groups (Figure 5E).

## Discussion

Breast cancer is a malignant tumor that threatens women’s health. There are approximately 1.3 million newly diagnosed breast cancer cases every year in the world, and nearly 500,000 people die of breast cancer every year [15,16]. Recently, the treatment of breast cancer has improved, and the treatment method has also evolved from a single surgical treatment to a comprehensive treatment with surgical resection, supplemented by chemotherapy, endocrine therapy, and molecular targeted therapy [17]. ‘Individualized treatment’ has become the new guiding principle for clinical work, but approximately 30% of breast cancer patients will still have recurrence and metastasis after comprehensive systemic treatment [18]. In some breast cancer patients who have already metastasized at the time of initial diagnoses, traditional chemotherapeutic drugs have obvious effects at first, but most patients will relapse and become resistant after a period of time [19]. Although the use of chemical drugs can significantly improve the survival rate of breast cancer patients, 80% of patients will develop resistance to varying degrees [20]. In particular, triple-negative breast cancer progresses rapidly and has a poor prognosis. Except for traditional chemotherapy, endocrine and molecular targeted therapy cannot be performed. Therefore, the development of new targeted molecules is an urgent issue for researchers.

Recently, miRNAs have been reported to affect the regulations of many human diseases, such as digestive system disease, metabolic disease, cardiovascular disease, inflammatory diseases, and numerous types of cancers [21,22]. Numerous reports have shown that miR-221/222 are involved in many physiological processes including cell proliferation, differentiation and apoptosis, as well as in several types of human cancers with diverse effects [23]. In the present study, we first determined the high expression levels of miR-221/222 in breast cancer tissues compared with its normal adjacent tissues and evaluated their anti-apoptotic factors in breast cancer cells. The results suggested that the miR-221/222 might play an important role in breast carcinogenesis. We next looked for target genes of miR-221/222 and identified GAS5 as a co-target, which plays a pivotal tumor suppression role in the occurrence and development of various cancers. The results indicated that combined miR-221/222 overexpression may be involved in the progression of breast cancer through co-targeting tumor suppressor GAS5 in this malignancy. In future studies, we predict identification of transcription factors that can potentially regulate miR-221/222. We also found that silencing GAS5 expression using siRNA could inhibit the apoptosis of breast cancer cells, whereas overexpressing GAS5 had a remarkable effect in promoting cell apoptosis. Notably, we identified the direct inhibition of GAS5 by miR-221/222 using a luciferase reporter assay. Furthermore, because miR-221/222 and GAS5 had opposing effects on cell apoptosis, it is possible that miR-221/222 suppressed GAS5 expression and consequently inhibited cell apoptosis, and then promoted tumor growth during breast cancer progression. We also showed that the restoration of GAS5 expression successfully attenuated the anti-apoptotic effects of miR-221/222 on breast cancer cells, indicating that the targeting of GAS5 may be a major mechanism through which miR-221/222 exerted its anti-apoptotic function.

At present, the correction of cellular miRNA levels has emerged as a potential therapeutic strategy for a wide range of diseases from genetic disorders to cancers and viral infections [24]. Overexpression of miRNAs can be silenced using antagomirs, and re-expression of miRNAs that are lost in diseases can be expressed by the overexpression of miRNA mimics [25]. With the advancement of nanotechnology, miRNA-based therapeutics can lead to more medical breakthroughs, which may revolutionize the treatment of diseases.

In summary, we not only identified the critical roles of miR-221/222 as oncomiRs in breast cancer, but also characterized the molecular mechanisms through which miR-221/222 contributed to breast cancer progression and identified GAS5 as a direct target gene. The regulation of GAS5 by miR-221/222 may explain why the up-regulation of miR-221/222 during breast carcinogenesis promotes tumor growth. Taken together, the present study characterized the molecular mechanism of breast carcinogenesis and provided new options for its treatment.

## Abbreviations

GAS5: growth arrest–specific transcript 5
H&E: hematoxylin and eosin
lncRNA: long non-coding RNA
